# Synergistic effect between LH and estrogen in the acceleration of cumulus expansion via GPR30 and EGFR pathways

**DOI:** 10.18632/aging.104029

**Published:** 2020-10-28

**Authors:** Jie Liu, Ru Yao, Sihai Lu, Rui Xu, Hui Zhang, Juncai Wei, Chunrui Zhao, Yaju Tang, Chan Li, Haokun Liu, Xiaoe Zhao, Qiang Wei, Baohua Ma

**Affiliations:** 1 College of Veterinary Medicine, Northwest A&F University, Yangling 712100 Shaanxi, China; 2 Key Laboratory of Animal Biotechnology, Ministry of Agriculture, Yangling 712100, Shaanxi, China

**Keywords:** LH, 17β-E_2_, GPR30, EGFR, cumulus expansion

## Abstract

The estrogen membrane receptor GPR30 (also known as G-protein coupled receptor 30) has recently been shown to be involved in the regulation of oocyte maturation and cumulus expansion. However, whether GPR30 expression is regulated by gonadotropin stimulation and how it participates in the regulation of the maturation process is still not clear. In this study, we explored the mechanism underlying the synergy between luteinizing hormone and 17β-estradiol (17β-E_2_) to improve the epidermal growth factor (EGF) response in cumulus oocyte complexes (COCs) during oocyte maturation in mice. The expression and distribution of GPR30, EGFR, and EGF-like growth factors were examined by real-time quantitative PCR, western blot, and immunofluorescence staining. Lyso-Tracker Red labeling was performed to detect the lysosomal activity in follicle granular cells (FGCs). Cumulus expansion of COCs was evaluated after in vitro maturation for 16 h. We found that EGF-like growth factors transmit LH signals to increase GRP30 levels by inhibiting protein degradation in lysosomes. Meanwhile, 17β-E_2_ stimulates the GPR30 signaling pathway to increase EGF receptor levels, enhancing the response ability of EGF signaling in COCs and thus promoting cumulus expansion. In conclusion, our study reveals the synergistic mechanism between LH and estrogen in the regulation of cumulus expansion during oocyte maturation process.

## INTRODUCTION

Estrogens are the primary sex hormones in female mammals, which play crucial roles in controlling the functions of reproductive system [1]. The main forms of estrogen are estrone (E_1_), estradiol (E_2_), and estriol (E_3_), of which E_2_ is the most active form in premenopausal women [2]. It has been proven that E_2_ promotes epithelial cell proliferation in the uterine endometrium and mammary glands [3]. Moreover, E_2_ produced by the placenta is related to the preparation for milk production during pregnancy [4]. Estrogen exerts its biological function through receptors, and two types of estrogen receptors have been reported in previous studies: nuclear receptors (ERs, including ERα and ERβ) and the membrane receptor GPR30 [5]. ERs are demonstrated to have a direct effect on the regulation of gene expression by binding to DNA sequences [1], but GPR30 has always been reported to act independently of changes in gene expression [6]. In our recent study, GPR30 was shown to be involved in the progression of oocyte meiotic resumption via rapid close the gap-junction intercellular communication between cumulus cells and oocytes [7]. However, whether GPR30 participates in other processes of oocyte maturation is not clear.

In mammals, the pituitary gland releases the luteinizing hormone (LH) to trigger oocyte maturation and ovulation during sexual maturity. Multiple processes are initiated by the increased levels of LH, which include meiotic resumption, cumulus expansion, and steroidogenesis [8]. However, the receptor that responds to LH stimulation was not detected in both oocyte and cumulus cells during follicle development and ovulation, and cumulus oocyte complexes (COCs) failed to respond when directly exposed to LH *in vitro* [9]. These results indicated that the effect of LH on COCs was indirect. Researchers have found that LH rapidly increases the expression of epidermal growth factor (EGF) family members, including amphiregulin (AREG), epiregulin (EREG), and betacellulin (BTC) in mural granulosa cells, and these factors act as paracrine mediators transmitting LH signals to COCs [10].

In the present study, we demonstrated the physiological mechanisms underlying the synergism between LH and 17β-E_2_ in the acceleration of cumulus expansion. Briefly, the GPR30 protein accumulates in cumulus cells in response to the LH signal; meanwhile, EGFR is upregulated via the GPR30 signaling pathway, which is stimulated by 17β-E_2_ to accelerate cumulus expansion. This finding helps us to better understand the function of estrogen in the process of oocyte maturation.

## RESULTS

### GPR30 protein accumulated in COCs after LH/hCG injection in mice

To detect the expression pattern of GPR30 in COCs during the process of oocyte maturation *in vivo*, PMSG-primed female mice were stimulated intraperitoneally with hCG, and the COCs were collected from ovaries at 0, 2, 4, 8, and 16 h. The mRNA and protein levels of GPR30 were measured. We found that although the mRNA levels of *GPR30* had rapidly decreased after hCG injection (Figure 1A), interestingly, the GPR30 protein accumulated in COCs over time (Figure 1B, 1C). These results suggest a negative feedback might exist in COCs that accumulation of GPR30 protein decrease *GPR30* transcription.

**Figure 1:** **GPR30 protein accumulated in COCs after LH/hCG injection. PMSG-primed female mice were injected with hCG, and the COCs in the ovaries were collected at 0, 2, 4, 8, and 16 h. The mRNA levels of *GPR30* were measured using RT-qPCR.** (**A**) The protein levels of GPR30 were detected using western blot (**B**), and the bands were quantified using gray scanning (**C**). Data are represented as fold induction relative to the unstimulated control (0 h). The bars of panels **A** and **C** are represented as average±SEM. Different lowercase letters indicate significant differences among the different groups (*p*<0.05). Three independent replicates were performed for each experiment.

### EGF-like growth factors transmit LH/hCG signals to induce GPR30 accumulation in COCs

To investigate whether the expression of EGF-like growth factors is stimulated by LH/hCG, mouse ovaries were collected to detect the mRNA levels of *AREG*, *EREG,* and *BTC* after hCG injection. The results were in line with previous research, as the mRNA of EGF-like growth factors had sharply increased within 1 h [10]. Furthermore, although *AREG* mRNA levels rapidly decreased back to the original level, *EREG* and *BTC* amounts peaked at the fourth hour of stimulation and remained at relatively high levels for up to 16 h (Figure 2A–2C).

**Figure 2:** **EGF-like growth factors stimulated by LH/hCG, induced the accumulation of GPR30 protein in COCs.** PMSG-primed female mice were injected with hCG, and the ovaries were collected at 0, 2, 4, 8, and 16 h. The mRNA levels of *AREG* (**A**), *EREG* (**B**) and *BTC* (**C**) were measured using RT-qPCR. To further conform the role of EGF-like growth factors in LH/hCG–induced GPR30 accumulation in COCs, AREG (100 nM), EREG (100 nM), BTC (100 nM) and EGF (10 ng/mL) were added to the medium and COCs were cultured *in vitro*. *GPR30* mRNA levels was measured using RT-qPCR (**D**), the protein levels were detected using western blot (**E**) and the bands were quantified using gray scanning (**F**). Data are represented as fold induction relative to the unstimulated control (0 h or con). Bars are presented as average±SEM. Different lowercase letters indicate significant differences between groups (*p*<0.05). Three independent replicates were performed for each experiment.

To confirm the role of EGF-like growth factors in GPR30 protein accumulation in COCs, mouse COCs were cultured *in vitro* with or without AREG, EREG, BTC, or EGF for 8 h. The results showed that compared with unstimulated control, *GPR30* mRNA levels were significantly declined about 40~50% (*p<*0.05, Figure 2D), but GPR30 protein had significantly accumulated in COCs following treatment with all four growth factors (*p<*0.05, Figure 2E, 2F).

### EGF downregulates *GPR30* expression but induces accumulation of the protein in COCs

As previously reported, mural granulosa cells respond to stimulation with LH to release EGF-like growth factors [10]. In this study, 10 ng/mL EGF was used to mimic the LH surge in COCs during oocyte maturation *in vitro*. When COCs were cultured without EGF (control), *GPR30* mRNA levels significantly increased within 2 h and remained at a high level for up to 16 h (*p<*0.05), However, the mRNA levels of *GPR30* were significantly lower in the EGF treatment groups then in the controls at each time point (*p<*0.05 Figure 3A). In contrast to the mRNA levels, a constant increase in the GPR30 protein levels were observed in the EGF treatment groups (Figure 3B, 3C). Although there was a limited increase in the GPR30 protein levels during the maturation process in the control group, it was significantly lower than that observed in the EGF group at the same time point (*p<*0.05 Figure 3D, 3E).

**Figure 3:** **EGF downregulates the expression but causes protein accumulation of GPR30 in COCs cultured *in vitro.*** COCs isolated from PMSG-primed mice were treated with or without EGF for 0, 2, 4, 8, and 16 h. After that, *GPR30* mRNA levels were measured using RT-qPCR (**A**). The amount of GPR30 protein in COCs cultured with EGF was detected using western blot (**B**), and the bands were quantified using gray scanning (**C**). COCs were cultured in vitro with or without EGF for 8 and 16 h, GPR30 protein levels were detected using western blots (**D**), and the bands were quantified using gray scanning (**E**). Data are represented as fold induction relative to the unstimulated control (0 h) in panels (**A**), (**C**) and (**E**), and bars are presented as average±SEM. In panels **A** and **E**, “*” indicated that *p<*0.05, and “**” indicated that *p<*0.01. In panel **C**, different lowercase letters indicate significant differences between groups (*p<*0.05). Three independent replicates were performed for each experiment.

### LH/EGF promotes GPR30 protein accumulation via a non-genomic pathway mediated by the activation of EGF receptor

To investigate whether the accumulation of GPR30 in COCs is regulated by the EGFR signaling pathway, AG1478 (an EGFR tyrosine kinase inhibitor) was used to block the activation of EGFR. In the *in vivo* experiment, as shown in Figure 4, mice were treated with AG1478 (1 mg/kg body weight, dissolved in saline with 15% captisol) or captisol (control) by intraperitoneal injection every other day (48 h interval), and PMSG was injected after the third dose. Then, hCG (or saline) was injected 48 h later. After that, COCs were collected 8 h later. The results showed that hCG significantly activated p-EGFR (Tyr1068), but AG1478 blocked the activation of p-EGFR induced by hCG stimulation (*p<*0.05). Moreover, GPR30 protein levels increased after hCG injection, but decreased by AG1478 treatment (*p<*0.05, Figure 5A, 5B).

**Figure 4:** **Illustration of mice treatment. In the control group, mice were intraperitoneally injected with captisol (dissolved in saline) on days 1, 3, 5, and 7, and PMSG was injected on day 5.** Saline was injected on day 7, COCs were collected on day 8. In the hCG group, all treatments were the same as for the control group, except that hCG was injected in mice instead of saline. In the AG1478 group, mice were treated with AG1478 on days 1, 3, 5, and 7, and PMSG was injected on day 5. hCG was then injected on day 7, and COCs were collected on day 8.

**Figure 5:** **LH/EGF promoted GPR30 protein accumulation in cumulus cells via a non-genomic pathway mediated by the activation of the EGF receptor.** Mice were treated as shown in Figure 4, The proteins were detected using western blot (**A**), and the bands of GPR30 were quantified using gray scanning (**B**). PMSG-primed mice received EGF or EGF plus AG1478 (AG) for 8 h, proteins were detected by western blot (**C**) and the bands of GPR30 were quantified using gray scanning (**D**), the mRNA levels of *GPR30* were measured using RT-qPCR (**E**). Immunostaining showed the fluorescence intensity (**F**) and the distribution (**G**) of GPR30 in the control, EGF, and EGF plus AG1478 groups, bar=50 μm. The amount of EGFR in COCs was detected by western blot (**H** and **I**), OOs indicate the oocytes and CCs indicate the cumulus cells. Data are presented as fold induction relative to the unstimulated control (con). Bars are presented as average±SEM. Different lowercase letters indicate significant differences between groups (*p*<0.05). Three independent replicates were performed for each experiment.

In the *in vitro* experiment, GPR30 protein levels was significantly increased by EGF treatment, accompanied with p-EGFR (Tyr1068) activation (*p<*0.05). However, the accumulation of GPR30 protein was downregulated when p-EGFR was blocked by 3 μM AG1478 (*p<*0.05, Figure 5C, 5D). Moreover, as mentioned above, the mRNA of *GPR30* was downregulated by EGF stimulation, while AG1478 reversed the inhibition of GPR30 transcription caused by EGF treatment (*p<*0.05, Figure 5E).

### LH/EGF promotes GPR30 accumulation in cumulus cells but not in oocytes

A cumulus oocyte complex consists of an oocyte (OO) and cumulus cells (CCs) that surround it. We analyzed the difference in GPR30 accumulation between oocyte and cumulus cells using immunofluorescence staining. The results revealed that EGF stimulation significantly promoted the accumulation of GPR30 in cumulus cells, but AG1478 reversed the accumulation caused by EGF treatment (*p<*0.05, Figure 5F, 5G). However, little change in intensity was observed in oocytes in the control, EGF, and EGF plus AG1478 groups (*p>*0.05, Figure 5F, 5G). To further confirm the relationship between EGFR activation and GPR30 accumulation, the distribution of EGFR in COCs was studied. The results showed that EGFR was mainly located in cumulus cells, and only to a small extent in oocytes (Figure 5H, 5I), which indicated that the LH/EGF-mediated increase in GPR30 protein levels primarily occurred in cumulus cells.

### Activated EGFR positively regulates GPR30 protein stability

Because of the limited number of cumulus cells, primary follicle granular cells (FGCs) were used for further experiments. Initially, COCs were treated with EGF or EGF plus AG1478, and protein expression was detected. The results showed that, similar to cumulus cells, GPR30 protein had also accumulated in FGCs after EGFR activation (Figure 6A–6C).

**Figure 6:** **EGFR positively regulates GPR30 protein stability.** Primary FGCs were treated with EGF to determine whether GPR30 accumulated after EGFR activity. (**A**) Western blot of proteins in FGCs after EGF treatment. (**B**) Graphical representation of the quantification of GPR30 protein levels shown in panel **A**. (**C**) Immunolabeling of the FGCs with GPR30 antibody (green) and DAPI (blue), bar=10 μm. (**D**) Western blot of GPR30 in FGCs treated with CHX only. (**E**) Western blot of GPR30 in FGCs treated with CHX plus EGF. (**F**) Graphical representation of the quantification of GPR30 protein levels shown in panels **D** (con) and **E** (EGF) to determine protein half-life. Data are presented as fold induction relative to the unstimulated control (0 h). The bars of panels **B** and **F** are presented as average±SEM. Different lowercase letters indicate significant differences between groups (*p*<0.05). Three independent replicates were performed for each experiment.

As shown in Figure 3A, EGF downregulates *GPR30* gene expression in COCs. Thus, we questioned why the level of GPR30 protein was increased after EGF treatment. For this purpose, the stability of GPR30 protein was assessed using the translational inhibitor cycloheximide (CHX, 50 μg/mL). Adherent FGCs (with or without 10 ng/mL EGF addition) were subjected to CHX for 0 to 5 h, followed by western blot analyses. In the control group, the protein mass of GPR30 was significantly decreased in the second hour of CHX treatment (Figure 6D). However, in the EGF group, the effect of CHX on GPR30 protein mass was significantly delayed (Figure 6E). Through intensity analysis, we found that the half-life of the GPR30 protein in the control group was approximately 2 h, but it was extended to more than 5 h when EGFR was activated (Figure 6F).

### Activation of EGFR maintains GPR30 protein stability by reducing the quantity and inhibiting the activity of lysosomes

The lysosomal and ubiquitin-proteasome pathways are two major routes for intracellular protein degradation. To study the pathway involved in GPR30 degradation, FGCs were treated with the lysosome inhibitor bafilomycin A1 (BA1, 500 nM) and the proteasome inhibitor MG132 (10 μM) for 4 h, and the same dose of DMSO was added to the control group. As shown in Figure 7A and 7B, GPR30 protein mass was higher in the BA1-treated group (lane 2) than in the control (lane 1) and MG132-treated (lane 3) groups (*p<*0.05). LC3 is an autophagy-related protein that was used as an indicator of lysosomal activity in the current study. The accumulation of LC3 protein in the BA1 group indicated that the concentration of BA1 was effective (Figure 7A). Previous reports demonstrated that the EGFR was degraded through both the lysosomal and ubiquitin-proteasome pathways [11, 12]. In this study, the accumulation of EGFR protein in the MG132 group indicated that the dose of MG132 was effective in FGCs (Figure 7A). These results indicated that GPR30 was mainly degraded through the lysosomal pathway in FGCs.

**Figure 7:** **The GPR30 protein is degraded via the lysosomal pathway.** FGCs were treated with the lysosome inhibitor BA1 or proteasome inhibitor MG132 (MG) for 4 h, GPR30 was detected using Western blot (**A**), and the quantification of GPR30 protein levels are shown in the diagram (**B**). Data are presented as fold induction relative to the unstimulated control. Bars are presented as the average±SEM. Different lowercase letters indicate significant differences between groups (*p*<0.05). Three independent replicates were performed for each experiment.

Furthermore, lysosome activity was detected in FGCs with and without EGF treatment. As shown in Figure 8A, the activity of lysosomes decreased after EGF treatment when compared with the control. In the next experiment, GPR30 and LAMP1 (a membrane protein located at the surface of the lysosome, used to indicate the quantity of lysosomes in cells) co-localized in FGCs. As shown in Figure 8B, the fluorescence of GPR30 was stronger in the EGF group then in the control. On the contrary, the fluorescence of LAMP1 was weaker in the EGF group than in the control. These results indicated that less lysosomes were present in FGCs after EGF treatment, and the activity of lysosomes was inhibited by EGFR activation.

**Figure 8:** **The activity and quantity of lysosomes were both downregulated by EGF treatment in FGCs.** Lysosomal activity was detected by Lyso-Tracker red, bar=50 μm (**A**). The quantity of lysosomes was evaluated by immunostaining (**B**), GPR30 antibody (red), LAMP1 antibody (green), and DAPI (blue), shown in this panel, bar=10 μm. “Neg” indicates negative control (secondary antibodies only). Three independent replicates were performed for each experiment.

### GPR30 activation increases EGFR protein levels in COCs

Interestingly, we found that the EGFR protein levels in COCs continually increased until 8 h after hCG injection *in vivo* (Figure 9A, 9B). However, EGFR levels rapidly decreased when EGFR was activated in COCs cultured *in vitro* (Figure 9C, 9D). In this case, we hypothesized that estrogen in follicles may play a role in maintaining or even increasing the EGFR levels in COCs. The results showed that EGFR protein levels were significantly higher in the medium containing 17β-E_2_ (1 μM) than in the control (*p*<0.05). To ascertain which estrogen signaling pathway participates in the regulation of EGFR, G1 (1 μM, a high-affinity, selective agonist of GPR30), G15 (1 μM, an antagonist of GPR30), and ICI182780 (1 μM, an antagonist of ERs) were added to the culture medium, and EGFR protein levels were detected by western blot. As shown in Figure 9E and 9F, EGFR levels were significantly increased by 17β-E_2_ or G1 addition in COCs. However, combined 17β-E_2_ and G15 treatment significantly decreased the EGFR levels. Moreover, ICI182780 addition could not reverse the increase in EGFR caused by 17β-E_2_.

**Figure 9:** **EGFR protein was increased by GPR30 activation in COCs.**PMSG-primed female mice were injected with hCG, and the COCs in the ovaries were collected at 0, 2, 4, 8, and 16 h. After that, the EGFR protein levels were evaluated using western blot (**A**) and quantified using gray scanning (**B**). COCs were cultured *in vitro* with EGF treatment for 0, 2, 4, 8, and 16 h, EGFR protein was detected using western blot (**C**) and quantified using gray scanning (**D**). In the next experiment, 17β-E_2_, G1, G15 and ICI182780 were used to explore the mechanism of estrogen in the maintenance or even upregulation of EGFR levels in COCs cultured *in vitro* for 8 h. EGFR protein levels were detected using western blot (**E**) and quantified using gray scanning (**F**). Data are represented as fold induction relative to the unstimulated control (0 h or con). Bars are presented as average±SEM. Different lowercase letters indicate significant differences between groups (*p*<0.05). Three independent replicates were performed for each experiment.

### The E_2_/GPR30 pathway enhances the response to EGF and accelerates cumulus expansion

COCs were collected from ovaries and cultured for 16 h, after which, the cumulus expansion index was evaluated. As shown in Figure 10, the cumulus could not expand without EGF treatment, not only in the control group, but also in the 17β-E_2_ or G1-treated groups. Furthermore, cumulus expansion was significantly induced by 1 ng/mL EGF, and a higher level of expansion was observed in the group treated with 10 ng/mL EGF. However, 1 ng/mL EGF plus 17β-E_2_ or G1 significantly increased the expansion index and the number of grade 4 COCs compared with 1 ng/mL EGF alone (*p<*0.05). Moreover, G15, but not ICI182780, significantly reversed the increase in the cumulus expansion index induced by 17β-E_2_ (*p<*0.05).

**Figure 10:** **The E_2_/GPR30 pathway enhances the response of EGF signaling and accelerates cumulus expansion.** COCs were cultured in the medium with 1 ng/mL EGF, 10 ng/mL EGF, 17β-E_2_, G1, G15 or ICI182780 addition for 16 h, and the cumulus expansion level was assessed. (**A**) Representative images of COCs isolated from ovaries (0 h) and cultured under different conditions for 16 h. (**B**) CEI of COCs cultured for 16 h in each group. (**C**) The different grades of COC culture for 16 h in each group. Data are represented as average±SEM. Different lowercase letters indicate significant differences (*p*<0.05). Three independent replicates were performed for this experiment.

### The E_2_/GPR30 pathway positively regulates the expression of cumulus expansion-related genes *HAS2*, *PTGS2* and *TNFAIP6*

Next, the expression of cumulus expansion-related genes *HAS2*, *PTGS2*, *TNFAIP6* and *PTX3* was detected. The results showed that, compared with the 1 ng/mL EGF group, 1ng/mL EGF plus 17β-E_2_ or G1 significantly increased the mRNA levels of *Has2, PTGS2* and *TNFAIP6* in COCs (*p<*0.05), G15, but not ICI182780, significantly reversed the increase in mRNA levels of these genes (*p<*0.05). In addition, neither 17β-E_2_ nor G1 could upregulate the expression of *HAS2*, *PTGS2*, *TNFAIP6* or *PTX3* without EGF treatment (Figure 11).

**Figure 11:** **E_2_/GPR30 signal activation upregulates cumulus expansion-related genes in the presence of EGF.** COCs were cultured in the medium with 1 ng/mL EGF, 10 ng/mL EGF, 17β-E_2_, G1, G15 or ICI182780 for 8 h, and the cumulus expansion-related genes (*HAS2, PTGS2, TNFAIP3* and *PTX3*) were detected using RT-qPCR. Data are represented as fold induction over unstimulated control. Bars are represented as average±SEM. Different lowercase letters indicate significant differences between groups (*p<*0.05). Three independent replicates were performed for each experiment.

## DISCUSSION

### LH triggers increased GPR30 protein in cumulus cells by inhibiting the quantity and activity of lysosomes via the EGFR signaling pathway

It is widely accepted that LH is an essential hormone that regulates oocyte maturation in mammals. In each reproductive cycle, ovaries receive the LH signal, and the oocytes within preovulatory follicles resume meiosis, followed by maturation and ovulation [13]. In this process, LH induces a series of changes in the theca and granulosa cells (such as reprogramming of gene expression or changes in secretory properties) to promote the maturation and acquisition of developmental competence in oocytes [14, 15]. In the current study, we found that the GPR30 protein in granulosa cells (including CCs and FGCs) continued to accumulate after hCG/EGF exposure, implying that GPR30 might participate in the process of oocyte maturation. However, the *GPR30* mRNA levels in granulosa cells decreased after hCG/EGF treatment, and a similar expression pattern was observed in the ovary of hamsters [16]. Therefore, we assume that some negative feedback exists that downregulates *GPR30* expression upon GPR30 protein accumulation in cells in an attempt to maintain the GPR30 protein at an acceptable level.

Due to the lack of the LH receptor in cumulus cells and oocytes, the effect of LH-induced oocyte maturation and cumulus expansion depends on the paracrine effect of mural granulosa cells. EGF-like growth factor family members AREG, EREG, and BTC are rapidly expressed in mural granulosa cells after the LH surge [10]. Activation of the EGFR network in COCs is essential for ovulation through multiple signaling cascades, including a decrease in the amount of CNP in follicles [17], phosphorylation and activation of cGMP phosphodiesterase PDE5 in oocytes [18], dephosphorylation and inactivation of NPR2 in cumulus cells [19], and promotion of the expression of cumulus expansion-related genes [10]. In this study, the accumulation of GPR30 protein in granulosa cells was inhibited by AG1478 treatment, which demonstrated that the EGFR network also participates in the regulation of GPR30 levels.

The results indicated that the EGF signal could not upregulate *GPR30* transcription, so we considered that GPR30 protein accumulation might be caused by an obstacle in degradation processes. The lysosomal and ubiquitin-proteasome systems are two major intracellular pathways for protein degradation [20, 21]. Many studies have demonstrated that GPR30 is degraded via the ubiquitin-proteasome pathway in HEK293 cells [22–24]. However, we found that proteasome inhibitor MG132 treatment could not induce the accumulation of GPR30 in FGCs. Nevertheless, the lysosome inhibitor bafilomycin A1 protected GPR30 from degradation. The difference suggests that different metabolic pathways existed in different cell types. Furthermore, we demonstrate that activated EGFR not only decreased the number but also inhibits the activity of lysosomes in FGCs, which prolonged the half-life of GPR30 protein from 2 hours to over 5 hours.

### Activation of GPR30 increases EGFR levels and accelerates cumulus expansion in COCs developed *in vitro*

It was observed that GPR30 levels in granulosa cells responded to LH signaling. Therefore, we hypothesized that GPR30 play a role in oocyte maturation. It was previously shown that sustained EGFR activity is essential for oocyte maturation in preovulatory follicles [25], and the developmental competence of oocytes is improved by promotion the EGFR signal [26]. EGF signaling pathway is involved in a series of important cell processes, such as proliferation, differentiation, apoptosis, and cell motility. Thus the activity of the EGFR is tightly regulated [27, 28]. EGF binding to its receptor activates the associated tyrosine kinase via phosphorylation, which results in the stimulation of numerous signaling cascades. In parallel, phosphorylated EGFR is internalized by clathrin-mediated endocytosis and thus deactivated [29]. Internalized p-EGFR passes through the early endosome and late endosome, dephosphorylated, and is finally delivered for degradation or recycling back to the membrane [30]. Maintaining adequate EGFR levels on the membrane is important to sustain EGFR activity during oocyte maturation. In this study, a significant difference in EGFR levels was found between the *in vivo* and *in vitro* experiments, which implies that the EGFR levels are regulated by some other mechanism in the ovary follicle. Estrogen is mainly synthesized in the ovary [31], and in the current study, we demonstrated that estrogen is involved in the regulation of EGFR levels via the GPR30 signaling pathway.

The EGF network is critical for cumulus expansion during oocyte maturation [32, 33], and the absence or immaturity of EGFR causes low developmental competence in COCs [26]. It was also reported that COCs developed *in vitro* with 17β-E_2_ exhibited increased levels of cumulus expansion and *HAS2* transcription compared to those developed without 17β-E_2_ [34]. However, in this experiment, we found that although the addition of 17β-E_2_ or G1 helped to accelerate cumulus expansion and cumulus expansion-related gene (*HAS2*, *PTGS2* and *TNFAIP6*) expression, this effect was not observed under the separate activation of GPR30 without the participation of EGF signaling. Likewise, the expression of cumulus expansion-related genes was not upregulated by 17β-E_2_ or G1 treatment individually. Furthermore, we demonstrate that the activation of GPR30 promotes the EGF response in COCs exposed to lower concentrations of EGF. These results indicate that estrogen increases EGFR levels in COCs by activating GPR30 signaling pathway, which helps COCs respond better to EGF stimulation.

In conclusion, during mouse COC maturation, LH positively stimulates GPR30 production in cumulus cells by activation of the EGFR pathway and the inhibition of lysosomes. In parallel, estrogen increases the EGFR levels to accelerate cumulus expansion by promoting the response to EGF signals in COCs via the GPR30 signaling pathway (Figure 12).

**Figure 12:** **Schematic of mechanisms by which LH synergy with estradiol accelerates cumulus expansion during oocyte maturation in mice.**

## MATERIALS AND METHODS

### Reagents

All chemicals were purchased from Sigma-Aldrich (MO, USA), unless specified otherwise. LH was purchased from Sansheng Biological Technology (Ningbo, China). Recombinant human amphiregulin, recombinant human epiregulin and recombinant human betacellulin were purchased from PeproTech (NJ, USA). AG1478 was purchased from Abmole Bioscience (TX, USA). Cycloheximide was purchased from Apexbio Technology (TX, USA).

### Animals

Female Kunming mice (approximately 4 weeks old) were used in all experiments. The mice were obtained from the Air Force Medical University of People’s Liberation Army of China, maintained on a 12 h light/dark cycle, and fed with food and water *ad libitum*.

### Ethics approval

All procedures described in this research were reviewed and approved by the Institutional Animal Care and Use Committee of the College of Veterinary Medicine, Northwest A&F University (No. 2018011212).

### COCs collection

For *in vivo* COC collection, mice were intraperitoneally stimulated with 5 IU of PMSG, followed by 5 IU hCG 48 h later, and were then sacrificed by cervical dislocation at 0, 2, 4, 8, and 16 h after hCG injection. In the 0, 2, 4, and 8 h groups, COCs were collected from antral follicles in the ovaries, and in the 16 h group, the COCs were collected from oviducts.

For *in vitro* COC collection, mice were intraperitoneally stimulated with 5 IU of PMSG, and 46-48 h later, mice were sacrificed, and ovaries were collected under sterile conditions. After that, COCs (250-350 μm in diameter) were collected from antral follicles. COCs containing compact cumulus cells were used for experiments. Minimum Essential Medium Alpha (MEM-α) containing Glutamine (Life Technology, CA, USA) and supplemented with 0.3% bovine serum albumin (BSA) was used as the culture medium.

### Isolation and culture of follicle granular cells

Mice were intraperitoneally stimulated with 5 IU of PMSG, and 46-48 h later, ovaries were collected and moved to 35 mm dishes filled with 2 mL MEM-α. Then, the antral follicles were punctured to release COCs and FGCs. The tissues and COCs were removed, and other liquids were collected and centrifuged for 5 min at a speed of 1000 rpm. The cells were collected at the bottom of centrifuge tubes and washed within PBS three times. After that, cells were resuspended in DMEM/F12 (Life Technology) containing 10% FBS in dishes, and the dishes were placed in a 37.0 °C, 5% CO_2_ incubator. Cells were washed three times in PBS 24 h later to remove red blood cells, and the FGCs were kept adherent to the dishes. Finally, FGCs were cultured in DMEM/F12 in an incubator for another 24 h in order to reach 70-80% confluence, and the cells were used for experiments.

### RNA extraction and quantitative reverse transcription polymerase chain reaction (RT-qPCR) analysis

Total RNA in Tissues and COCs was extracted using the MiniBEST Universal RNA Extraction Kit (Takara, Tokyo, Japan) and then reverse transcribed to produce complementary DNA (cDNA) with PrimeScript™ RT Master Mix (Takara) following the manufacturer's instructions. RT-qPCR analysis was used to measure the expression levels of genes encoding *GPR30*, *EGFR*, *AREG*, *EREG*, *BTC*, *HAS2*, *PTGS2*, *PTX3*, *TNFAIP6,* and *GAPDH* (as an internal control). The RT-qPCR assay was performed using TB Green^®^ Premix Ex Taq™ II (Takara). The amplification conditions were as follows: template denaturation and polymerase activation at 95 °C for 1 min, followed by 40 cycles of amplification at 95 °C for 5 s, and annealing at 60 °C for 34 s. The data are representative of three independent assays, and the levels of mRNA were calculated using the 2^−ΔΔCT^ method. The specific primers designed are listed in Table 1.

**Table 1:** Primers sequences of target genes and the reaction conditions.

**Gene name**	**Primer sequences forward (F) and reverse (R)**	**Amplicon size (bp)**	**NCBI Reference Sequence**
GAPDH	F: 5’-TCACTGCCACCCAGAAGA-3’	185	XM_017321385.2
	R: 5’-GACGGACACATTGGGGGTAG-3’		
GPR30	F: 5’-CCTCTACACCATCTTCCTCTTTC-3’	109	XM_006504757.4
	R: 5’-GATGAAGTACAGGTCTGGGATG-3’		
EGFR	F: 5’-ACTGCTGCCACAACCAATGTGC-3’	92	XM_029483270.1
	R: 5’-GCATGTGGCCTCATCTTGGAAC-3’		
AREG	F: 5’-TGCCTAGCTGAGGACAATGC-3’	126	NM_009704.4
	R: 5’-AGTGACAACTGGGCATCTGG-3’		
EREG	F: 5’-CTTGGGAGGTGTCTGCAAGT-3’	133	NM_007950.2
	R: 5’-AACCACTGTGCCAAGCCATA-3’		
BTC	F: 5’-GCCCTGGGTCTTGCAATTCT-3’	150	NM_007568.5
	R: 5’-GCACCGAGAGAAGTGGGTTT-3’		
HAS2	F: 5’-AAGACCCTATGGTTGGAGGTGTT-3’	167	NM_008216.3
	R: 5’-CATTCCCAGAGGACCGCTTAT-3’		
PTGS2	F: 5’-CCCTTCCTCCCGTAGCAGAT-3’	111	NM_011198.4
	R: 5’-TGAACTCTCTCCGTAGAAGAACCTTT-3’		
PTX3	F: 5’-GGGCTCAAACTCGGATCACT-3’	133	NM_008987.3
	R: 5’-GAGGTCTCAGCCACTACTGC-3’		
TNFAIP6	F: 5’-ATACAAGCTCACCTACGCCGAA-3’	123	NM_009398.2
	R: 5’-ATCCATCCAGCAGCACAGACAT-3’		

### Western blot analysis

Western blot was performed as described previously [7]. Cells or COCs were lysed in RIPA buffer supplemented with 1 mM PMSF (Solarbio, Beijing, China) and were kept on ice for 10 min. The protein concentration was determined using the BCA method. After that, protein was denatured with SDS-loading buffer in a 100 °C metal bath for 10 min, Equal amounts of the protein from each group were loaded onto 10% SDS-PAGE gels, and were then transferred to PVDF membranes (Millipore, MA, USA). The membranes were blocked in TBST supplemented with 5% skim milk powder (BD, NJ, USA) for 1.5 h and incubated with primary antibodies at 4 °C overnight. After three washes in TBST, the membranes were incubated with HRP-conjugated goat anti-rabbit IgG (Sangon Biotech, Shanghai, China) at 4 °C for 12 h. The membranes were washed three times in TBST, the blots were visualized with a chemiluminescent HRP substrate reagent (Bio-Rad Laboratories, CA, USA), and images were acquired using a chemiluminescence system Tanon-5200 (Tanon Science & Technology Co. Ltd, Shanghai, China). Antibodies against GAPDH (#2118, 1:2000 dilution), and Phospho-EGF Receptor (Tyr1068, #3777, 1:2000 dilution) were purchased from CST (Cell Signaling Technology, MA, USA). Antibodies against GPR30 (ab39742, 1:2000 dilution), EGFR (ab32077, 1:2000 dilution) and LC3 (ab51520, 1:8000 dilution) were purchased from Abcam Limited (Cambridge, UK). The primary antibodies were diluted in the Primary Antibody Dilution Buffer (Solarbio), The HRP-conjugated Goat Anti-Rabbit IgG (D110058, 1:5000 diluted in TBST) was purchased from Sangon Biotech (Shanghai, China). The images shown are representative of at least three independent experiments.

### Immunofluorescence staining

Samples (COCs or FGCs) were fixed in 4 % paraformaldehyde (Solarbio) for 2 h in room temperature (RT, approximate to 25 °C), permeabilized in PBS containing 0.1% Triton X-100 for 10 min at RT, and were then blocked in PBS containing 3% BSA for 2 h. The fixed and permeabilized samples were incubated with goat GPR30 antibody (Abcam, ab118512) and/or rabbit LAMP-1 antibody (Proteintech, IL, USA, 55273-1) at a dilution of 1:200 in PBS containing 3% FBS overnight at 4 °C. The target proteins were visualized by incubating with secondary antibodies of Alexa Fluor 488-labeled donkey anti-goat (Abcam, 150129), Alexa Fluor 594-labeled donkey anti-goat (Abcam, ab150132), or Alexa Fluor 488-labeled donkey anti rabbit (Life Technologies, # A-21206) at a dilution of 1:300 at RT for 2 h in the dark. After incubation with antibodies, the nuclei of samples were stained with DAPI (10 μg/mL) for 5 min at RT. The samples were washed with PBS three times after each step. After staining, the samples were mounted on slides, and the slides were observed under a confocal scanning laser microscope (Nikon Eclipse Ti, Tokyo, Japan). Images shown are representative of at least three independent experiments.

### Lyso-Tracker Red staining

The lysosomal activity of FGCs with or without EGF treatment was analyzed by Lyso-Tracker Red (Beyotime, Shanghai, China) according to the manufacturer's instructions. Briefly, Lyso-Tracker Red was diluted in culture medium at a concentration of 50 nM and preincubated at 37 °C for 15 min. Then, the warmed Lyso-Tracker Red medium was used to label the cells for 60 min at 37 °C. The nuclei were labeled by 10 μg/mL DAPI for 3 min at RT. After that, the solution was replaced with fresh culture medium, and the cells were photographed using a fluorescence microscope (Olympus IX71, Tokyo, Japan).

### COCs expansion assay

COCs collected *in vitro* were allowed to undergo IVM for 16 h under different conditions, and the cumulus expansion index (CEI) was calculated following the formula described by Fagbohun and Downs [35].

### Statistical analysis

All experiments were performed with at least three independent replicates. The relative mRNA and protein levels of GPR30 in COCs with or without EGF treatment for same exposure time (Figure 3A and 3E) were analyzed by the Student’s t-tests, and other data were analyzed by one-way ANOVA followed by the Duncan’s multiple comparison test using the software SPSS Statistics 19.0. The results are presented as mean ± SEM. *p<*0.05 was considered statistically significant.
